This article has been retracted.

# Analysis of Sino-Russian Media Cooperation and the Construction of International Online Public Opinion Discourse under the Dual Influence of Ecological and Online Environments

**DOI:** 10.1155/2022/7740313

**Published:** 2022-08-17

**Authors:** Juxi Zhang, Chongyu Ma

**Affiliations:** ^1^School of Journalism and Communication, Zhengzhou University, Zhengzhou 450001, China; ^2^Foreign Studies College, Hunan Normal University, Changsha 410081, China

## Abstract

In the context of traditional media, the media can dominate the topic and composition of public opinion, but in the context of the convergence of online media, the dominance of public opinion has gradually evolved from the direction of the coexistence of single items and pluralism, especially from the international level. In other words, the construction of the comprehensive strategic writing partnership between China and Russia in the new era has given a new orientation and connotation to the bilateral relations and cooperation in the new era. In the face of an increasingly complex international public opinion environment, media cooperation between China and Russia is crucial. Therefore, based on an in-depth analysis of the construction of the discourse power of international public opinion under the dual influence of the ecological environment and the network environment, the construction of the discourse power of international public opinion is discussed from the aspects of the construction of discourse objects, the construction of the main body, and the enrichment of the content of international communication.

## 1. Introduction

At the present stage, the development of media integration under the network environment has gradually formed an information communication channel with online newspapers, radio, and television as the main body [1]. With the support of network media, the transmission speed of information has been further improved, and people's access to information is more and more convenient. The huge information cluster can also meet the personalized needs of the audience. At the same time, it also indirectly has a certain impact on the guidance of public opinion of network media. Of course, the development of network media has also brought new changes to international communication. The in-depth development of social media has indirectly promoted the transformation and reconstruction of the right to speak. International communication has undergone great changes in media selection, actors, communication mode, communication content, and influence. Multimedia, rich and diversified video content presentation, and other forms of network television have gradually become an important position of international communication [2]. The construction of the comprehensive strategic writing partnership between China and Russia in the new era has given a new positioning and connotation to the bilateral relations and cooperation in the new era. In the face of the increasingly complex international public opinion environment under the network environment, the media of China and Russia must continue to deepen cooperation and jointly occur on international and regional issues, so as to better reflect the responsibility spirit and strategic cooperation effect of the two countries in order to build the voice of international public opinion [3, 4].  Figure 1 shows the theoretical model of the generation of the discourse power of international public opinion in the network environment.

The basic viewpoints of ecological environment are adaptation viewpoint, selection viewpoint, holistic viewpoint, hierarchy viewpoint, dynamic viewpoint, evolution viewpoint, and synergy viewpoint. In more than 100-year history of ecological development, ecological environment research has gone beyond the scope of biology. Ecosystem is to use the concept of ecology to explain the relationship between organizations and the environment. All the mutual influence and interaction between enterprise organizations and individuals rely on their respective core capabilities to complement each other's advantages to achieve common realization. The complex economic groups formed by value innovation belong to the enterprise ecosystem. Ecosystems are interdependent and interact with their environment. With the emergence of computer networks and changes in the network environment, the traditional business model of organizations has undergone tremendous changes, and the impact of the environment on the organization has also expanded. The network environment is composed of technical and social aspects. The network ecological environment situation analysis can be customized. Network ecological purification requires an overall analysis of situational data. Situational awareness can be introduced into the analysis engine in the form of a plug-in, so that the analysis engine can be customized according to different business needs, and the analysis engine can be customized to make the special rectification of network ecology purification more effective and efficient. The future trend of the network ecological environment is predictable. One of the functions of situational awareness systems is forecasting, so forecasting models are introduced. In the network ecological environment, for the collected network ecological big data, through machine learning, the introduction of prediction models can better predict the future network ecology, provide support for decision-making, and reduce the occurrence of extreme network events.

## 2. Literature Review

For the theory of discourse power, many scholars have systematically expounded Foucault's theory of discourse and power to a certain extent and combed the relationship between discourse and power from a philosophical point of view. Some scholars define the concept of dialogue right from Habermas' communicative behavior theory and discourse politics theory. Some scholars start with Foucault's theory of discourse power, pointing out that the function of “discourse” is “empowerment.” Some scholars elaborate on the connotation of dialogue right and international discourse right and put forward that only having discourse right can guide public opinion to develop in the direction beneficial to our side. Some start with the theory of ancient Chinese philosophy, expound the connotation, essence, and function of discourse, and emphasize the important role of discourse in the field of public opinion [5, 6].

According to the theory of international discourse power, some scholars have explained and defined the international discourse power from the perspective of international politics. Some explained in detail what is the right to speak, why our party should attach great importance to the right to speak, how to have the right to speak, and how to expand and strengthen the right to speak. Some scholars elaborated on the ideological transformation in China's diplomacy and the changes, main construction directions, and tasks of new China's diplomatic discourse. By analyzing the current international situation of international discourse power, some scholars put forward the opportunity of improving China's international discourse power. From the perspective of the community of shared future of mankind, some scholars analyze the definition of international discourse power by three main theoretical schools: power discourse power from the perspective of realism, institutional discourse power from the perspective of Neo liberal institutionalism, and development discourse power from the perspective of dependency theory. Some scholars put forward how to lead the promotion of China's international discourse power by building a community with a shared future for mankind. Some analyze the construction path of China's international discourse right from the construction task and concept of China's international discourse right in the new era. Based on the definition of international discourse power by three main theoretical schools, some scholars pointed out the current situation of imbalance, disorder, and anomie of the international discourse power system and put forward a Chinese plan for global governance of international discourse power reform from the perspective of a community of shared future for mankind [7, 8].

In the research of public opinion discourse power, scholars mostly discuss it from the perspective of discourse power theory or the news thought of Chinese state leaders. Some scholars have explained the discourse power and influence of media public opinion, pointed out that the discourse power and influence of media public opinion complement each other, and summarized the problems and countermeasures in the use of media public opinion discourse power. Some scholars have discussed the connotation of the discourse power of public opinion from the perspective of discourse power and proposed to expand and strengthen the discourse power from multiple perspectives. Some scholars emphasize that news communication should first pay attention to the right of discourse, strengthen the awareness of the right of discourse, and exercise the right of discourse of the media. Some scholars emphasize that the core of public opinion guidance lies in the competition for the right to speak, think that the main elements of the right to speak are the right to speak, the right to spread, and the right to guide, and put forward a new path of public opinion guidance. Some scholars pointed out that news and public opinion are an important carrier for a political party to master the right to speak [9]. The discourse power of news public opinion should obey certain political needs and guide the trend of news public opinion. Some scholars focus their research on how to reconstruct the discourse power of public opinion in the context of strategic communication and put forward five reconstruction paths to give full play to the strategic communication mechanism.

Thus, the academic research on the guidance of public opinion and the discourse power of public opinion focuses on two focal points: one is the research on the theory of “discourse power” of public opinion, and the other is the research on how to compete for the discourse power of public opinion. To sum up, most scholars believe that the focus and core of the guiding power of public opinion and the discourse power of public opinion are “discourse power.” Only by recognizing the importance of “discourse power” can we achieve due development in the exercise and competition of discourse power.

## 3. Analysis of the Foundation and Current Situation of the Construction of the Right to Speak of International Public Opinion under the Dual Influence of the Ecological Environment and the Network Environment

### 3.1. Take the Initiative to Open Up and Win Wide Public Opinion

In the face of the complex and changeable situation in today's world, China has gradually embarked on the road of active diplomacy and active opening-up, striving to create a new diplomatic situation and strive for the recognition of the international community. China adheres to the diplomatic strategy of “periphery is the primary, major countries are the key and developing countries are the foundation.” Fifth, China actively promotes and improves the development of relations with other countries and adheres to being good with its neighbors, seeking common ground while reserving differences and peaceful coexistence. Apart from a few countries that have cracks with China due to problems left over by history or other bad intentions, China maintains friendly relations with most countries. At the diplomatic level, China-Russia comprehensive strategic partnership enables the two countries to support each other and further maintain the peaceful ties of bilateral relations. China-EU relations have generally maintained stable development, and there are common contradictions based on common interests. At the same time, China actively carries out multilateral diplomacy, participates in the settlement of international hot issues, takes the initiative to assist countries with relatively backward development, and assumes the international responsibility of a big country [10, 11]. In recent years, the Chinese concept of the “the Belt and Road” and the “community of shared future for mankind” has won the attention of relevant countries since it was put forward. Through this, the international community has seen China's determination and sincerity to regard the people of the world as one and contribute to the overall development of all countries, nations, and the world. In terms of media cooperation, after officially establishing diplomatic relations with other countries, China has conducted multilateral exchanges with other countries in the field of journalism. By carrying out different degrees of exchange activities with countries with diplomatic relations in the fields of newspapers, book publishing, news, radio, and television, we can build an external communication system for other countries [12]. At present, Xinhua news agency, international radio and CCTV, and other media have achieved landing and localized production in many countries.

After years of diplomatic activities and media exchanges, China has strengthened its relations with other countries through a new situation of good diplomacy, which has won the recognition and support of the international community, especially the recognition of the majority of developing countries. Overall, China's peaceful and friendly diplomatic activities over the years have shaped the image of a responsible big country in front of the people of the world and won the basis of public opinion for itself. China is no longer isolated in the international community, nor will it allow the western media to misread our information and attack us by public opinion [13, 14].

In recent years, the proportion of China's GDP in the world's GDP has increased year by year. At present, China has jumped to the second place in the world and become a booster of world economic growth. In 2007, China's contribution rate to world economic growth surpassed that of the United States for the first time, becoming the first in the world. Today, many international economies are deeply benefited by China's economic development and have closer ties with China's economy. Economic growth has promoted the rapid development of other areas of the country, increased economic investment in science and technology, military, national defense, and other fields, and effectively promoted the steady improvement of the country's overall strength.  Table 1 shows the GDP ranking of countries in the world in 2019.

Although countries have long recognized the inequality and imbalance of the international discourse pattern and deeply understood the importance of the right to speak and the initiative, the actual situation has rarely been changed. After the 1990s, China's ability to influence the world has gradually increased, “hard power” drives “soft power,” and China's discourse expression has gradually been accepted and recognized by the international community, which is mainly reflected in two aspects [15].

First, foreign media pay close attention to China. The in-depth development of globalization, the rapid renewal of information technology, and the impact of China's increasingly powerful comprehensive national strength on the world have all made foreign media pay unprecedented attention to China. The early reports of Western media on China were mainly political issues, and there were many negative reports [16]. Since the new century, with the understanding of China, especially with the continuous improvement of the news opening and news release system, the increasing Chinese reports by Western media have become more and more close to the reality of China, and the balanced reports are increasing.

Secondly, the voice from China is gradually accepted. As a developing and emerging country, with the enhancement of its comprehensive national strength and the improvement of its international status, especially the expansion of the international influence of the development model of socialism with Chinese characteristics, China has objectively posed an impact and challenge to the value system, development model, and even acceptance psychology of the western world, which is difficult for those who have long occupied the dominant position to accept calmly and willingly. We should pursue the victory and realize the international recognition of our due voice of international public opinion to the greatest extent in the process of promoting the reform and reconstruction of international voice, which is related to the long-term interests and development in the future.

### 3.2. Analysis on the Current Situation of the Construction of the Discourse Power of International Public Opinion from the Perspective of New Media

The visual culture represented by ubiquitous and all-time online video is occupying the world. Video services under the names of video portals, video websites, and online TV stations are becoming the focus of global Internet applications, social attention, and the development of radio and television. Since 2017, the “TikTok” short video has become popular all over the world. By 2019, its overseas version of “TikTok” has been implemented in 75 languages in 150 countries around the world. By the first quarter of 2020, TikTok's global total downloads exceeded 2 billion (regardless of the third-party Android platforms in China and other regions), and the downloads of app store and Google play in a single quarter exceeded 300 million, making it the mobile application with the highest downloads in the world (see Figure 2). TikTok enriches and disseminates short video content from a global perspective through the access of localized content in various regions. It is a successful case of “going global” mobile short video application.

#### 3.2.1. The Main Object of Discourse Construction of International Public Opinion

*(1) First, Distribution by Region*. According to the region of the audience, we can divide the audience of international public opinion into China and foreign countries. Foreign audiences can be divided into western countries and nonwestern countries. In terms of audience division between China and foreign countries, mainstream media often spread to audiences outside China by setting up different media platforms [17]. For example, the “people's network” of the people's Daily has a Chinese version and an overseas version, respectively, which realizes the synchronization of the content dissemination of the same media for different audiences.  Table 2 shows the distribution of Xinhua news agency abroad:

*(2) Second, Distribution by Media*. Taking people's daily and people.com as examples, for different paper and online media, there are clear differences in the choice of discourse objects between them (see Table 3). Secondly, emerging media, such as search engine represented by Baidu, news client represented by Tencent News, social media represented by WeChat, and short video media represented by TikTok, have very different audience choices due to their different communication characteristics and modes (see Table 4).

#### 3.2.2. Audience Orientation of China's International Public Opinion Discourse

Influenced by the multiple factors of “personalization” and “socialization” of network users, the new network media take more account of the autonomy and differentiation of the audience and fully understand the uncontrollable characteristics of the network audience in the process of international public opinion guidance. For example, the target audience set by “People's Network” is different from that of “People's Daily” (see Table 5).

In terms of information dissemination, although Xinhua News Agency shoulders the important task of external communication of official mainstream media, it not only focuses on a certain region, but also broadens its vision to the global scope and transmits information in an all-round way. Xinhua news agency has not only set up hundreds of branches around the world; moreover, on the new online media, it has opened Chinese and foreign language websites at the same time and opened an official account on the global social media platform. See Tables 6 and 7.

CGTN China International Television (global television network) is under the command of Beijing headquarters, including the global operation of overseas regional production centers, reporter stations, and other dispatched agencies in various languages. It has six TV channels in English, Spanish, French, Arabic, Russian, and records, a video news agency and a new media cluster dominated by mobile news networks. It has implemented the whole channel or some programs in more than 170 countries and regions around the world. Previously, the number of fans of CGTN's official Facebook account exceeded 100 million, becoming the largest news media in the world. The YouTube account has more than 300 million news video hits, ranking first among the central media. CGTN new media cluster has become one of the main channels for international audiences to understand China.  Table 8 shows the number of major media websites in China.

Through the classified statistics of news topics (taking the English version of people's network as an example, see Table 9), and through the proportion of Politics (policy, democracy, diplomacy, etc.), economy, culture (education, tradition, etc.), society (people's livelihood, disaster, etc.), science, technology, environmental protection, and health in the reports, we can see the distribution of news topics of “people's network.” Among the 70 news reports, there are 30 political news, 18 economic news, 4 cultural news, 6 social news, and 12 science, technology, sanitation, and agriculture news. Among them, political news and economic news account for the largest proportion, accounting for 43% and 25.7%, respectively. It is worth mentioning that, in the political and diplomatic relations reports, the reports on China US relations account for almost half of such reports, which is the most common topic in the news reports reflecting China US relations. In addition, because the third Import Trade Expo is in progress during this period, there are also 6 news items on the theme of the Expo.

As can be seen from Table 10, among the 70 headline news reports on the front page of the English version of renmin.com, there are 49 stories featuring China, accounting for 70% of the total sample, 9 stories featuring “China + other countries,” accounting for 12.9%, and international news accounting for 2.8%, with only 2 stories. It can be said that news reports with China as the protagonist or with direct interests with China account for 86% of the total news, nearly nine-tenths of the total. And less than one-fifth of all news reports focus on other countries, including 9 in the United States, accounting for 90% of the news of “other countries,” with the highest proportion.

In the era of new media on the Internet, the news sources of the media are no longer single, and they are interviewed, edited, and released by their own journalists. They have more diversified news sources [18]. As the official mainstream media news website, the English version of renmin.com mainly comes from authoritative news media. Among the 70 news reports, 42 were from Xinhua news agency, accounting for 60%, ranking first. The news from People's Daily and People's Network was 11 and 11, respectively, accounting for 15.75%. In addition, there are 3 news stories from China Daily, 2 news stories from Global Times, and 1 news story from CGTN. See Figure 3 for source analysis.

It is analyzed from two aspects, that is, news theme and reporting tendency, reporting protagonist and reporting tendency. The first is the news theme and reporting tendency. From Table 11, there are 21 positive tendency reports, including 6 political news, 6 economic news, 4 science and technology news, 1 social livelihood news, and 1 culture, environmental protection, health, and agriculture news. From Table 12, among the reports with negative tendency, 6 are political news, 1 is economic news, and 1 is cultural news.

From the perspective of the relationship between the reporting protagonist and the reporting tendency, in the positive reports, there are as many as 18 with China as the reporting protagonist and 3 with “China + other countries” as the reporting protagonist. In this way, all positive reports are either dominated by China or have direct interests with China. Among the negative tendency reports, there are 4 reports on China US relations, including “decoupling between China and the United States is bad for everyone,” “persecution of Chinese journalists by the United States,” “American interference in Hong Kong,” and “American political bullying”; there are 4 reports with the United States as the protagonist, involving American politics, economy, and culture [19].

From the perspective of media brand communication power, the communication power of central news media websites in overseas social media platforms is shown in Table 13. The highest communication power of each platform is as follows: Xinhua ranks the highest in the communication power of Google and twitter, China Radio Network (CNR) ranks the highest in the communication power of Wikipedia, People's Network ranks the highest in the communication power of Facebook, and China Daily ranks the highest in the communication power of Instagram.

In terms of audience size, after years of audience accumulation, China's news media have formed a considerable number of audience groups (see Table 14). China's influential traditional mainstream media, relying on rich funds, advanced technology, policies, talents, and other resources, continue to improve themselves in external communication, and most of their English news websites have strong communication power overseas.

After information circulates in the international public opinion market, it will produce short-term or long-term, expected or unexpected diversified communication effects, including the impact and results on the general audience, news media, or other media institutions of other countries and the international community. Through the guidance of media public opinion, discourse communication acts on people's cognition and behavior system, which will produce corresponding discourse effects and cause changes in people's cognitive institutions, value system, emotional attitude, and behavior to a certain extent, involving multiple levels such as cognition, attitude, and action, so as to obtain the effect feedback from the audience [20]. Whether the audience effect feedback meets the communication expectations of the discourse subject is directly related to the effect of communication activities, which reflects the discourse influence of a country's media.

## 4. The Construction of the Discourse Power of International Public Opinion under Sino-Russian Media Cooperation under the Dual Influence of Ecological Environment and Network Environment

### 4.1. Based on the High Political Mutual Trust and Close Interest Ties between the Two Sides

First of all, the Chinese and Russian media should adhere to “content is king,” strengthen in-depth news cooperation, and improve the ability of setting the international agenda. With the popularity of the Internet, the ways for the audience to obtain information are increasing, and the problem of excess information is becoming more and more prominent. Chinese and Russian media should continue to enhance the public reliability of news gathering and editing, highlight authoritative views and voices, and create “the first source of information” and “the first right of interpretation” in a large amount of information. Through opinion guidance and public opinion guidance, the audience can better understand the changes of the objective situation. The media of the two countries need to further increase the dimension and thickness of their reports on each other. They should not only actively voice in international issues dominated by themselves or involving each other, but also coordinate with each other in the reporting of major events related to the world political pattern [21]. After the “law revision storm” in Hong Kong in 2019, the special report “uncover the mask of Hong Kong” launched by “Russia today (RT)” has aroused widespread concern in the international community. The report focused on the behind the scenes of the situation in Hong Kong, unveiled the “figure of Washington” under the mask, and was considered by the majority of netizens to have issued a “voice of justice,” which has become an example of the coordinated voice of the media of the two countries to influence international public opinion.

Secondly, in the context of media convergence, the two sides should break through the mindset, actively create highlights of cooperation in the field of new media, and contribute wisdom to international cyberspace governance. With the in-depth integration and development of media, the boundary between traditional TV media and emerging media has become blurred. The definition and competition for the field of public opinion are also gradually changing. Today, there is no need to “deliberately divide mass communication and interpersonal communication, audience scene and user scene, people's oral public opinion field, and mainstream media public opinion field. As long as there are people, groups, circles, and social places and platforms that can produce effective communication and influence, they should take the initiative.” Therefore, relying on the good cooperation of traditional media, China and Russia should actively explore a wider range of linkage platforms including PC, app, and social networking. As a new media exchange platform of “resource accommodation, content integration, mutual publicity, and interests' integration,” the “China Russia headline client” is one of the fruits of the continuous cooperation between the media of the two countries in line with the development of the times. The client was jointly built by the former China Radio International and the “Russia Today” international news agency, which gathered the advantageous resources of the mainstream media, fully took care of the needs of both audiences, and achieved good communication results. At present, China and Russia are constantly exploring cooperation paths of mass collection, multiple generation, and multiple communication, in order to realize resource sharing and complementary advantages in the field of new media. On the basis of the platform, the media should make full use of the cross-border, cross time, and even cross language characteristics of network communication, focus on the commanding heights and key points of global issues, the hotspots, and highlights of friendly exchanges between the two countries, work together to create high-quality content, open up communication channels, and jointly expand their influence in the international public opinion field and cyberspace [22]. In particular, the global public field in which netizens share and discuss international affairs in the social network scene should be fully considered. At present, the number of Internet users in China and Russia is nearly 1 billion, which is the backbone of the Internet public opinion field. According to the attributes and characteristics of social communication, Chinese and Russian media should occupy the voice of civil networks by jointly holding activities, creating “opinion leaders” and other flexible ways.

### 4.2. Strengthen Technical Exchanges and Cooperation and Enable Content Production and Influence Formation through Technological Innovation

New technologies and applications have revolutionized the media field and opened up new development space for content production. China and Russia are both big countries in the development of new media, with similar development background and foundation, such as rising industrial demand and strong technological *R*&*D* strength. Guided by advanced technology, the two sides should further promote the cooperation and layout of the media of the two countries in the fields of “5 g + 4 K/8 K + AI” and build a media technology innovation community. Both sides need to strengthen the research and application of new generation information technologies such as artificial intelligence, blockchain, 5G, and big data in the field of network communication, timely grasp new trends, and develop new products, so as to make technology the biggest support for the evolution and breakthrough of the Internet. The period from 2020 to 2021 is the “year of scientific and technological innovation between China and Russia,” jointly determined by the two heads of state, and media technical cooperation is its due meaning. Both sides should seize the favorable opportunity to strive for the transformation of media production mode and content form, so as to meet and occupy the needs of more users.

### 4.3. Make Full Use of Multilateral Cooperation Platforms to Enhance the Driving Force and Leadership of Chinese and Russian Media

China and Russia are not only members of the UN Security Council, but also carry out close cooperation under the framework of SCO, BRICs, and other international organizations. With the construction and docking of the “the Belt and Road” and the “Eurasian Economic Union,” the exchanges between the two countries and relevant countries along the line have been deepened. Today, with the rapid development of informatization and digitization, it is in the interests of all parties to effectively voice multilateral cooperation.

China and Russia should make full use of the media cooperation mechanism under the framework of relevant organizations to promote institutionalized and normalized practical cooperation between the media of Member States, strengthen exchanges and coordination, make use of each other's strength and voice together, and carry out news reporting cooperation on major regional and international issues [23]. Led by China and Russia, we will strengthen the establishment of an Internet cooperation mechanism among Member States, expand the integration and interaction of new media, finally realize the mutually beneficial and win-win situation of “cyberspace,” and promote the construction of a good public opinion environment and communication order [24, 25].

## 5. Conclusion

Under the dual influence of the ecological environment and the network environment, people are more free to express their views on social events and national political events through the network media. The views expressed by each person represent the venting of personal views, either rational, perceptual, objective, or subjective. The views expressed by each person represent the venting of personal views, either rational, perceptual, objective, or subjective, which will affect the voice of public opinion of online media. Some extreme, false, provocative, and even malicious attacks and abuse will often lead online media astray. Therefore, under the background of media integration, network media should take effective strategies to guide public opinion to the track of health and order in line with the mainstream values of society. In the field of international communication, behind the right to speak is the contest between the country's hard power, soft power, and the country's position in the global system. The “rise of other parts of the world” led by emerging countries led by China and Russia has become a major theme of world politics and economy in the 21st century. With the improvement of national comprehensive strength and influence, Chinese and Russian media should have a matching position in the world communication pattern. At the same time, in order to compete for national influence and maximize national interests, the media of the two countries need to give full play to their constructive role. Therefore, standing at the new historical starting point of China Russia relations and global governance pattern, the two sides should comply with and grasp the development trend of digital media, learn from each other, constantly expand the field of cooperation, innovate the content of cooperation, gradually enhance the influence of international public opinion, and promote the establishment of a new global media order.

## Figures and Tables

**Figure 1:** Theoretical model of the generation of discourse power of international public opinion under the network environment.

**Figure 2:** Global downloads of TikTok (unit: million times).

**Figure 3:** Distribution of headline news sources on the English version of People's Daily news website.

**Table 1:** Ranking of world GDP (2019).

Ranking	Name	GDP (USD, IMF' 2019)	GDP (USD, UN' 2016)	Per capita GDP	Population in 2019
1	America	21.34 trillion	18.62 trillion	$64866	329064917.00
2	China	14.22 trillion	11.22 trillion	$9916	1433783686.00
3	Japan	5.18 trillion	4.94 trillion	$40803	126860301.00
4	Germany	3.96 trillion	3.48 trillion	$47463	83517045.00
5	India	2.97 trillion	2.26 trillion	$2176	1366417.75
6	Britain	2.83 trillion	2.65 trillion	$41897	67530172.00
7	France	2.76 trillion	2.47 trillion	$4240	65129728.00
8	Italy	2.03 trillion	1.86 trillion	$3346	60550075.00
9	Brazil	1.96 trillion	1.80 trillion	$9239	211049527.00
9	Canada	1.74 trillion	1.53 trillion	$46487.00	37411047.00

**Table 2:** Regional distribution of Xinhua news Agency branches abroad.

Region	Asia pacific region	Eurasian region	Middle east	American region	African region
Quantity	22	23	19	19	19
Proportion	21.50%	22.50%	18.60%	18.60%	18.60%

**Table 3:** Audience selection of people's daily media in different media platforms.

	People's daily	People's network (news website)	Official microblog of people's daily	Official WeChat official account of people's daily
Audience range	Mainland readers, overseas Chinese and compatriots in Hong Kong, Macao and Taiwan, but excluding foreigners who do not understand Chinese.	There are random internet users who have internet habits all over the world and often browse the web page.	Internet users who are used to relying on microblog for information.	Network users who rely on WeChat official account to obtain information.
Characteristic	Fixed and single scope	Random and wide range	Younger and diversified	Multilevel and multiage

**Table 4:** Main audience groups of emerging media platforms.

	Media type	Target user	User scope
Baidu	Search engines	Ordinary netizens who need to collect information;	Global
Tencent news overseas edition	News website	Enterprise users who need to promote information collection.	Global
WeChat	Social media	A group that uses the internet to browse news content.	Global
TikTok	Short video social platform	Social media users	Global

**Table 5:** Comparison of audience positioning between “people's Daily” and “people's network.”

	People's Daily	People's Network
Audience range	Mainland readers, overseas Chinese and compatriots in Hong Kong, Macao and Taiwan, but excluding foreigners who do not understand Chinese.	Internet users who have the habit of surfing the internet and often browse the web page are random.
Audience age	Care about people over the age of 30 with mature political thought.	The age range is broad, but it is younger as a whole.
Audience professional structure	Mainly the staff of political party departments, government agencies, institutions and social organizations.	There is no obvious scope, and the occupational structure is complex, involving many fields such as politics, finance, science and technology.
Audience education level	With high cultural and educational background.	There are high or low education, with a large difference.
Audience social status	Generally high status in society.	Social status has both high and low, with a large gap.
Audience income level	Relatively stable income groups. The income gap between audiences is small.	Groups with relatively unstable income levels. The income gap of the audience is large

**Table 6:** Comparison of Chinese and foreign branches of Huashe.

	Branch	Total number of branches
China	33	53
Foreign country	102	180

**Table 7:** Comparison of Chinese and foreign social media official accounts opened by China news agency.

Platform set up	User scale	Platform set up	User scale
Sina Weibo	101.2 million (fans)	YouTube	103万
WeChat official account	20 million+ (fans)	Facebook	8752万
TikTok	35.62 million (fans)	Twitter	1259万

**Table 8:** Number of foreign language channels (websites) of major media websites in China.

Website	Number of foreign languages	Typical languages
Xinhuanet	7	English, Spanish, French, Russian, Arabic
People's network	6	English, Japanese, French, Spanish, Russian
China daily	2	English, French
International online	61	English, Japanese, French, Russian, German, Spanish
China network television	5	English, Spanish, French
Xinhuanet	7	English, Spanish, French, Russian, Arabic

**Table 9:** Distribution of headlines and news topics on the English version of Minwang news website.

Subject category	Detailed category	Quantity	Special remarks
Politics	China	15	Including China US diplomacy 4
	Other countries/International politics	6	
	Diplomatic relations	9	
Economics	Chinese economy	16	Including the expo 6
	World economy	2	
Culture	Chinese culture	3	
	Culture of other countries	1	
Sociology	China	5	
	International	1	
Technology and environmental protection	China	10	

**Table 10:** Distribution of protagonists in the headlines of the English version of the People's Daily news website.

Report protagonist		Quantity
China	China	49
	China + other countries	9

Other countries	USA	9
	Austria	1

International		2

**Table 11:** Positive tendency of headline news reports on the English version of People's Daily news website.

Theme	Report protagonist	Attitude keywords	Reporting tendency
Environment protection	China	High-quality, greener	Positive
Politics	China	Far-sighted	Positive
Politics diplomacy	China Finland	Thrive	Positive
Science and technology	China	Aided by technology	Positive
Politics diplomacy	Chinese/English	Recovery	Positive
Society people's livelihood	China	Improving	Positive
Politics	Hong Kong, China	Timely and essential	Positive
Agriculture	China	High yield	Positive
Economics	China	Help and stimulate consumption	Positive
Culture religion	China	Freedomfully	Positive
Economics	China	Pushes	Positive
Science and technology	China	Stronger momentum	Positive
Politics	China	Success	Positive
Technological innovation	China	New high	Positive
Politics diplomacy	China Finland	Friendly relation	Positive
Economics	China	Upward	Positive
Economics	China	sincerity, sense of responsibility	Positive
Science and technology	China	Remarkable performance	Positive
Economics	China	Provides impetus	Positive
Medical and health work	China	Promising	Positive
Economics	China	Growth	Positive

**Table 12:** Negative tendency of headlines on the English version of People's Daily news website.

Theme	Report protagonist	Attitude keywords	Reporting tendency
Politics diplomacy	China America	Unrealistic, harmful	Negative
Economics	America	Threaten	Negative
Culture	America	Threatens	Negative
Politics diplomacy	China America	Persecution, suppression	Negative
Politics diplomacy	China America	Meddling in	Negative
Politics	America	Deepeningdivide	Negative
Politics	America	Division, anxiety	Negative
Politics	America	Politicalbullying	Negative

**Table 13:** Ranking of communication power of foreign social media platforms of central news websites.

Platform ranking	Google	Wikipedia	Twitter	Facebook	Instagram
1	Xinhuanet	China broadcasting network	Xinhuanet	People's network	China daily
2	China news network	International online	People's network	China network television	China news network
3	Taiwan, China network	China daily	China daily	Xinhuanet	China Tibet online
4	China daily	China network television	China news network	China daily	Guangming net
5	International online	China news network	Guangming net	China net	International online

**Table 14:** Audience size of major social media platforms of Chinese media.

Media platform	Microblog (number of fans)	TikTok (number of fans)	YouTube (number of fans)	Facebook (number of fans)	Twitter (number of fans)
Xinhua news agency	100.28 million	35.689 million	1.02 million	87.52 million	12.569 million
China Daily	59.30 million	32.062 million	0.0356 million	103.612 million	4.347 million
People's Daily	123.17 million	12000 million	0.184 million	86.174 million	7.043 million
CRI international online	4.35 million	4.796 million	None	24.645 million	76.5 million
CGTN China international television	5.44 million	7.967 million	2.00 million	1.1257 million	13.724 million

## Data Availability

The labeled data set used to support the findings of this study is available from the corresponding author upon request.
